The article "Pakistan CO2 Emission Modelling and Forecasting: A Linear and Nonlinear Time Series Approach" was published in 2023. Journal: J Environ Public Health.

# Pakistan CO_2_ Emission Modelling and Forecasting: A Linear and Nonlinear Time Series Approach

**DOI:** 10.1155/2023/5903362

**Published:** 2023-01-31

**Authors:** Kassim Tawiah, Muhammad Daniyal, Moiz Qureshi

**Affiliations:** ^1^Department of Mathematics and Statistics, University of Energy and Natural Resources, Sunyani, Ghana; ^2^Department of Statistics and Actuarial Science, Kwame Nkrumah University of Science and Technology, Kumasi, Ghana; ^3^Department of Statistics, The Islamia University of Bahawalpur, Bahawalpur, Pakistan; ^4^Department of Statistics, Shaheed Benazir Bhutto University, Shaheed Benazirabad, Pakistan

## Abstract

Pakistan is considered among the top five countries with the highest CO_2_ emissions globally. This calls for pragmatic policy implementation by all stakeholders to bring finality to this alarming situation since it contributes greatly to global warming, thereby leading to climate change. This study is an attempt to make a comparative analysis of the linear time series models with nonlinear time series models to study CO_2_ emission data in Pakistan. These linear and nonlinear time series models were used to model and forecast future values of CO_2_ emissions for a short period. To assess and select the best model among these linear and nonlinear time series models, we used the root mean square error (RMSE) and the mean absolute error (MAE) as performance indicators. The outputs showed that the nonlinear machine learning models are the best among all other models, having the lowest RMSE and MAE values. Based on the forecasted value of the nonlinear machine learning neural network autoregressive model, Pakistan's CO_2_ emissions will be 1.048 metric tons per capita by 2028. The increasing trend in emissions is a frightening and clear warning, suggesting that innovative policies must be initiated to reduce the trend. We encourage the Pakistan government to price CO_2_ emissions by companies and entities per ton, adapt electricity production from hydro, wind, and different sources with no emissions of CO_2_, initiate rigorous planting of more trees in the populated areas of Pakistan as forest covers, provide incentives to companies, organisations, institutions, and households to come out with clean technologies or use technologies with no CO_2_ emissions or those with lower ones, and fund more studies to develop clean and innovative technologies with less or no CO_2_ emissions.

## 1. Introduction

The collection of greenhouse gas (GHG) emissions in airspace is creating chaos across the globe and destroying life, economy, health, and food. Carbon (IV) oxide (CO_2_) is a major component of GHG [1]. The world is nowhere near securing a global temperature rise of less than two degrees Celsius as proposed in the Paris Agreement of the United Nations (UN) Framework Convention on Climate Change (UNFCCC). Using the 1990 criterion, most countries are still releasing more GHG into the atmosphere, with some at a standstill and others releasing less [1]. The UN Environmental Program (UNEP) Climate Action Note indicated that the world is in a state of climate emergency [1].

The article "Pakistan CO2 Emission Modelling and Forecasting: A Linear and Nonlinear Time Series Approach" was published in 2023. Journal: J Environ Public Health.

Pakistan is labelled among the countries with the highest GHG emissions in the world by the UNEP [1]. It contributes to 1.02% of global GHG emissions. Pakistan emitted an estimated 504.59 million tons of GHG in 2018. It is one of the most impacted nations from unfriendly effects of environmental change as well as air contamination. GHG emissions are the leading cause of global warming, thereby becoming the maximum essential research issues within the fields of technological know-how and politics [1].

In Southern Asia, Pakistan is ranked among the developing economies with swift economic positive growth. This is expected to continue for a long time. Agriculture is the principal dominant area in Pakistan's economic growth irrespective of the growing industrial sector. However, this industrial drive, coupled with high population growth, has caused massive deforestation, resulting in less absorption of CO_2_ by plants, leading to a higher CO_2_ concentration in the atmosphere [2, 3].

Pakistan is ranked first among countries in Asia facing mass deforestation as a result of bulk utilization of natural energy from the environment. This is causing serious degradation of the environment. This degradation of the environment, together with deforestation, has brought about global warming, leading to climate change. The critical factor of Pakistan's commercial revolution is reworking its economy from organic economies based totally on human and animal energy to inorganic economies, which are completely dependent on fossil fuels. Interestingly, the by-product of fossil fuels is CO_2_, thereby contributing to the concentration of CO_2_ in the environment [2, 3].

The quest to be an industrialized giant definitely comes at a price. Pakistan is geared towards a full-industrial revolution which encourages the use of fossil fuels to power the growing industry in the country. The growth in population means expanding cities by destroying green vegetation, which absorbs most of the CO_2_ in the atmosphere. The growing population also means increasing cars with carbon emissions being used in the country [2, 3].

The Government of Pakistan has put in place a lot of programmes to reduce GHG emissions in the country. Great progress has been chalked up in climate action that ranges from policies, programmes, and nature-based solutions (NBS) to technology-based innovations [4]. Pakistan, recognizing the role of nature in climate modification and diminution, has put forward robust natural capital restoration plans including the Ten Billion Tree Tsunami Program as well as the Protected Drive. These programmes have contributed to enhancing livelihoods and giving opportunities to the vulnerable, including youth and women. In addition, Pakistan has introduced a number of policy actions focused on mitigating GHG emissions from high-emission sectors, such as energy and industry [4].

The article "Pakistan CO2 Emission Modelling and Forecasting: A Linear and Nonlinear Time Series Approach" was published in 2023. Journal: J Environ Public Health.

Notwithstanding, this available information indicates a rise in CO_2_ emissions in Pakistan. This needs to be scientifically substantiated and verified to assist the government to restrategize in an attempt to achieve the targeted goal in the fight of reducing these emissions in order to achieve the Paris Agreement of the UNFCCC. This study provides a statistical and machine learning framework to delve deep into the discourse of CO_2_ emissions in Pakistan from 1960 to 2018. It provides CO_2_ emission forecasts for future and possible policy initiatives and directions to combat this issue based on scientific results to meet the UNFCCC target.

### 1.1. Literature Review

The world is being confronted with significant difficulties connected with an unnatural weather change and discharge of ozone-depleting substances in large amounts. In 2017, energy businesses represented 46% of all CO_2_ discharges worldwide [5]. Bokde et al. [5] proposed two-time series disintegration techniques for transient determination of CO_2_ outflow with a bunch of cutting-edge models for a 48-hour skyline power market. By estimating benchmarks for France, they showed that their new technique has a mean outright rate blunder, that is, 25% lower than that of existing models. Furthermore, they illustrated the use of the conjecture for booking adaptable power utilization in Germany, Norway, Denmark, and Poland. Their results showed that booking an adaptable block of 4 hour of power utilization at a 24-hour stretch can on average diminish subsequent CO_2_ discharge in all countries [5].

The carbon exchanging market has turned into a powerful weapon in easing fossil fuel by-products in China, and carbon cost is at the centre of its activity. Thus, the carbon exchanging market fills in as an imperative part in gauging carbon cost precisely ahead of time [6]. Sun and Li [6] imaginatively investigated a group of driven long short-term memory network (LSTM) models in light of reciprocal outfit experimental mode decay (ROEMD) for carbon cost gauging, applying it to each of the eight carbon exchanging piloting centres in China. ROEMD was first executed for mode change to disintegrate the first convoluted mode into a bunch of straightforward modes. Accordingly, LSTM was utilized to demonstrate the planning between time-slacking factors and every model's objective quality, thereby constructing numerous LSTM models for comparison. At last, converse ROEMD computation was acquainted with the coordinates' expected consequences of the multimode on eventual outcomes. Its viable application at the same time embraced every one of the eight carbon piloting centres in China, covering their compared carbon cost information over a significantly extended period. The acquired outcomes showed that the proposed model had adequate precision in carbon cost anticipation in China in contrast to the single LSTM model as well as other ordinary machine learning models. Moreover, as indicated by the extent of its application, the creative model displayed solid dependability and comprehensiveness [6].

The article "Pakistan CO2 Emission Modelling and Forecasting: A Linear and Nonlinear Time Series Approach" was published in 2023. Journal: J Environ Public Health.

Wu and Liu [7] proposed a multiresolution combo-predicting model that uses ensemble empirical mode decomposition (EEMD-ADD) to improve the predicting accuracy of the cost of carbon. They achieved it by decomposing carbon price sequencing using EEMD into numerous intrinsic framework functions (IFFs) by dividing these IFFs into several high-frequency compartments, low-frequency compartments, and drift compartments after which the least square vector support machine (LSSVM), particle swarm optimization LSSVM (PSO-LSSVM), and bat algorithm-LSSVM (BA-LSSVM) were utilized to forecast three compartments, respectively. Similarly, Yun et al. [8] built a robust carbon price-predicting model of complete ensemble empirical mode decomposition with adaptive noise (CEEMDAN)-long short-term memory (LSTM) by blending the merits of CEEMDAN in decaying multiresolution time-frequency carbon price waves and the LSTM model by installing monetary waves.

A report by Eckstein et al. [9] positioned Pakistan as the fifth generally impacted country because of environmental changes throughout the course of recent years, while the author in [10] positioned Pakistan's air as the second generally contaminated in 2020. To diminish these effects, the nation needs to take broad variation and alleviation measures while changing the energy area towards dirtying and carbon impartial choices [11].

Existing studies imply that greater than two-thirds of GHG emissions in Pakistan come from fossil power-related CO_2_ emissions. Consequently, forecasting CO_2_ emissions is crucial for adjusting regulations to mitigate weather changes. The forecasting of CO_2_ emissions has been mentioned dramatically in [12].

The article "Pakistan CO2 Emission Modelling and Forecasting: A Linear and Nonlinear Time Series Approach" was published in 2023. Journal: J Environ Public Health.

Pao and Tsai [13] implemented the grey model to obtain CO_2_ emissions in Brazil between 1980 and 2007. A combination of models based on the optimization algorithms of quantum harmony and discounted mean square has been established and employed in CO_2_ emission forecasting for the world's top five countries with high CO_2_ emissions [14]. Auffhammer and Carson [15] came up with China's CO_2_ emission path using a set of panel data in a provincial-level framework [16–19]. The application of the traditional grey model and the upgraded grey model has been implemented to forecast CO_2_ emissions [20, 21].

From qualitative and quantitative perspectives, numerous discussions have been conducted on the relationship between consumption of energy, economic growth, and CO_2_ emissions [22]. Al-mulali and Sab [23] investigated the influence of the consumption of basic energy and emissions of CO_2_ on sixteen developing countries, focusing on the impact on the development of their economies. Wang et al. [24] examined the significant factors contributing to CO_2_ emissions in China's road freight transport. Zhang and Nian [25] computed the emissions of CO_2_ and examined the factors contributing to emissions in China's transport sector. In China, Lin et al. [26] developed a new bootstrap ARDL bounding test for CO_2_ emissions and industrial development. Pao and Tsai [27] conducted an examination of the dynamism of the causal relationship, linking the emission of pollutants, consumption of energy, and their output in Britain, Russia, India, China, and other countries over a definite period [28–34].

Little work has been conducted on providing mathematical and statistical modelling techniques for modelling and predicting CO_2_ emissions in Pakistan and where the country stands in the future concerning this important issue. It is against this backdrop that this paper provides a modelling and forecasting technique based on linear and nonlinear time series models. This study predicts the amount of CO_2_ emissions in Pakistan for almost a decade to assist the Pakistan government and other stakeholders to plan ahead to devise ways of mitigating the effects of CO_2_ emissions or possibly curtailing them.

Section 2 of the paper presents the source of data, data characteristics, and the modelling and forecasting techniques applied.  Section 3 presents the discussion and the results, while the last section presents the conclusions and recommendations of the study.

## 2. Materials and Methods

### 2.1. Data

The data are made up of CO_2_ emissions in Pakistan from 1960 to 2018. The amount of CO_2_ was measured in metric tons per capita according to international standards. The data were obtained from the World Bank data indicators of Pakistan (https://databank.worldbank.org/).  Figure 1 shows CO_2_ emissions (metrics tons per capita) from 1960 to 2018 as obtained from the World Bank. It can be observed from the figure that there is an increasing trend, which is an indication of a seasonal trend in the series. Seasonality must therefore be removed from the series before applying our modelling and forecasting techniques. The descriptive statistics in Table 1 show that the average CO_2_ emissions from 1960 to 2018 were 0.572 metric tons per capita, with a minimum CO_2_ emission of 0.314 metric tons per capita and a maximum of 0.981 metric tons per capita.

The article "Pakistan CO2 Emission Modelling and Forecasting: A Linear and Nonlinear Time Series Approach" was published in 2023. Journal: J Environ Public Health.

### 2.2. Methods

We present a brief outline of all linear and nonlinear time series models implemented in this study. In what follows, we illustrate the linear time series followed by nonlinear machine learning models.

#### 2.2.1. Linear Time Series Models

In this section, we give a brief outline of linear time series models, such as the Box–Jenkins ARIMA, trigonometric seasonality, Box–Cox transformation, ARMA errors, trend and seasonal model, naïve model, and exponential smoothing model.

*(1) Box–Jenkins ARIMA Modelling Approach*. The ARIMA (*p*, *d*, *q*) [35, 36] can be represented by

(1) $$\begin{array}{c} {\hat{X}}_{t}=\mu +\theta_{1}{\hat{x}}_{t-1}+\ldots +\theta_{p}{\hat{x}}_{t-p}+\ldots +\alpha_{1}e_{t-1}+\ldots +\alpha_{q}e_{t-q}+e_{t}\text{.} \end{array}$$

With lagged values $\theta_{1}{\hat{y}}_{t-1},\ldots ,\theta_{p}{\hat{y}}_{t-p}$ and lagged errors *α*_1_*e*_*t*−1_,…, *α*_*q*_*e*_*t*−*q*_. The *p*, *d*, and *q* of the series ${\hat{x}}_{t}$ are the autoregressive term order, the differencing degree of the series, and the moving average order term, respectively. The white noise *e*_*t*_ has mean 0 and variance *σ*^2^. The differencing of the series ${\hat{x}}_{t}$ can be conducted once or more times.

The seasonal multiplicative ARIMA model has the form ARIMA (*p*, *d*, *q*) × (*P*, *D*, *Q*) written as

(2) $$\begin{array}{c} \theta_{p}\left(K\right)\delta_{P}\left(E^{f}\right){\left(1-E\right)}^{d}{\left(1-E^{f}\right)}^{D}{\hat{X}}_{t}=∆+\vartheta_{q}\left(E\right)\mu_{Q}\left(E^{f}\right)\varepsilon_{t}\text{,} \end{array}$$

with *θ*_*p*_(*E*)=1 − *θ*_1_*E* − …*θ*_*p*_*E*^*p*^; *δ*_*P*_(*E*^*f*^)=1 − *δ*_1_*E*^*f*^ − …−*δ*_*P*_*E*^*Pf*^;  *ϑ*_*q*_(*K*)=1 − *ϑ*_1_*E* − …*ϑ*_*q*_*E*^*q*^;  an d *μ*_*Q*_(*E*^*f*^)=1 − *μ*_1_*K*^*f*^ − …−*μ*_*Q*_*E*^*Qf*^.

In the formula, *f* and *K* are the seasonality frequency and the shift balanced operator, respectively. The seasonal difference and ordinary differencing degrees are represented by *D* and d, respectively. *δ*_*P*_(*E*^*f*^)an d *θ*_*p*_(*E*) are the seasonal autoregressive polynomial of order *P* and regular autoregressive polynomial of order *p*, respectively while *μ*_*Q*_(*E*^*f*^)an d*ϑ*_*q*_(*E*) are the seasonal moving average of order *Q* and polynomials of the regular moving average of order *q*, respectively. Similarly, ∆ = *ρ*(1 − *θ*_1_ − …*θ*_*p*_)(1 − *δ*_1_ − …−*δ*_*P*_), where the mean of the process ${\left(1-E\right)}^{d}{\left(1-E^{f}\right)}^{D}{\hat{X}}_{t}$ is *ρ*. The white noise *ε*_*t*_ has mean 0 and variance *σ*^2^.

The article "Pakistan CO2 Emission Modelling and Forecasting: A Linear and Nonlinear Time Series Approach" was published in 2023. Journal: J Environ Public Health.

Figure 2 shows the diagrammatical display of the steps involved in this methodology. In Figure 2, it can be noticed that there are four steps involved in ARIMA modelling. We discuss the main steps involved in this method briefly.

**Step 1 .**

Identification of the ARIMA Model

This step requires the series to be stationary and parameters independent of time. In time series analysis, it is often found that the series is not white noised in advance. To make the series white noised, differencing is required. To test whether the series is stationary or not, we use the augmented Dickey–Fuller test. Once the series becomes stationary, graphical tools such as the autocorrelation function (ACF) and partial autocorrelation function (PACF) are implemented to identify the order of the candidate model.

**Step 2 .**

Model Estimation

With the help of the visual display of the autocorrelation function (ACF) and partial autocorrelation function (PACF) of the series, the appropriate candidate model for the series is estimated. Different combinations of candidate models are applied, and the final model is selected based on the criteria of accuracy of parameters.

**Step 3 .**

Diagnostic Checks

Here, the selected candidate model passes through various tests, which include the ACF plot, QQ-Norm plot, and Shapiro–Wilk to verify the normality of residuals. Once the model passes all these tests, the model is considered one of the best models for the next step.

**Step 4 .**

Forecasting

In this step, the candidate model fulfilling the three steps discussed earlier is used for predicting the future values of the series. The efficiency of the forecasted model is measured by the root mean square error (RMSE) and the mean absolute error (MAE). The mathematical expressions for RMSE and MAE are given by

(3) $$\begin{array}{c} \begin{array}{c} RMSE=\sqrt{\frac{1}{t-n}\overset{t}{\underset{i=n+1}{\sum }}{\left(x_{i}-{\hat{x}}_{i}\right)}^{2}},\\ MAE=\frac{1}{t-n}\overset{t}{\underset{i=N+1}{\sum }}\left|x_{i}-{\hat{x}}_{i}\right|\text{,} \end{array} \end{array}$$

where *x*_1_,…, *x*_*n*_ and *x*_*n*+1_,…, *x*_*t*_ are the partitions of the data for training and forecasting, respectively. In our case, we used the complete data for both training and forecasting. The RMSE and MAE assess the quality as well as summarize the model for superior forecasting. The model with the smallest RMSE and MAE values is chosen for forecasting [5]. Other indicators of measuring efficiency can also be implemented.

*(2) Trigonometric seasonality, Box-Cox transformation, ARMA errors, Trend, and Seasonal (TBATS) Modelling Approach*

The trigonometric seasonality, Box–Cox transformation, ARMA errors, trend, and seasonal component (TBATS) model is mainly used to predict the time series with complex seasonal patterns by exponential smoothing. The TBATS model utilizes the representation of trigonometric seasonal components based on the Fourier series. The TBATS model [38, 39] is given by

(4) $$\begin{array}{c} x_{t}^{\left(\alpha \right)}=\tau_{t-1}+\beta k_{t-1}+\overset{T}{\underset{i=1}{\sum }}\alpha_{t-n_{i}}^{\left(i\right)}+\vartheta_{t},\\ \tau_{t}=\tau_{t-1}+\beta k_{t-1}+\gamma \vartheta_{t},\\ k_{t}=\beta k_{t-1}+\omega \vartheta_{t},\\ \vartheta_{t}=\overset{p}{\underset{i=1}{\sum }}\;\delta_{i}\vartheta_{t-1}+\overset{q}{\underset{i=1}{\sum }}\theta_{i}\varepsilon_{t-1}+\varepsilon_{t}, \end{array}$$

where*x*_*t*_^(*α*)^ is the Box–Cox-transformed time series at moment *t* and *α*_*t*−*n*_*i*__^(*i*)^ is the *ith* seasonal component. *τ*_*t*_ is the local level, while *k*_*t*_ is the trend with damping. *ϑ*_*t*_ is ARMA (*p*, *q*) and *ε*_*t*_ is the white noise from a Gaussian process. *T* is the seasonality amount, whereas *n*_*i*_ is the length of the *ith* seasonal period. The Box–Cox transformation is *α*, while *β* is trending damping. Also, *ω*, *γ* represent the smoothing and *δ*_*i*_,*θ*_*i*_ are the ARMA (*p*, *q*) coefficients. *ε*_*t*_ is the white noise. The seasonal component of the TBATS model is given by

(5) $$\begin{array}{c} z_{t}^{\left(i\right)}=\overset{\left(l_{i}\right)}{\underset{i=1}{\sum }}z_{j,t}^{\left(i\right)}\;,\\ z_{j,t}^{\left(i\right)}=z_{j,t-1}^{\left(i\right)}\cos\left(\xi_{i}\right)+z_{j,t-1}^{*\left(i\right)}\sin\left(\xi_{i}\right)+\phi_{1}^{\left(i\right)}\vartheta_{t},\\ z_{j,t}^{*\left(i\right)}={-z}_{j,t-1}^{\left(i\right)}\sin\left(\xi_{i}\right)+z_{j,t-1}^{*\left(i\right)}\cos\left(\xi_{i}\right)+\phi_{2}^{\left(i\right)}\vartheta_{t}, \end{array}$$

where*ξ*_*i*_ = 2*πj*/*n*_*i*_ and *ϕ*_1_^(*i*)^, *ϕ*_2_^(*i*)^ are the seasonal smoothing.

*(3) Naïve Modelling Approach*. The naïve modelling approach utilizes the last year's genuine data as a figure for the current year. The following year's estimate *t*+1 will be equivalent to the current year's information [33]. The supposition that its interest lies later in the period will be equivalent to the interest in the last period. The expression of the naïve method [37, 40, 41] is

(6) $$\begin{array}{c} {\hat{X}}_{t+k}={\hat{X}}_{t}, \end{array}$$

The seasonal naïve model for the period *t*+*k* is of the form

(7) $$\begin{array}{c} {\hat{X}}_{t+k}={\hat{X}}_{t+k-n\left(g+1\right)}, \end{array}$$

where *n* is the period of seasonality and *g* is the integer part of *k* − 1/*n*, which is the number of years prior to the forecast year *t*+*k*.

*(4) Exponential Smoothing (ETS) Modelling Approach*. The exponential smoothing (ETS) technique is identically connected to one or more stochastic models. It likewise follows the property of robustness and treated as a model of critical extrapolation. The thought behind the ETS is that the estimates from this approach are the weighted normal average of past data, and weights exponentially decay with time. That is, the current data have bigger loads in contrast to the previous ones. In this way, ETS delivers savvy forecasting in contrast to typical techniques [37, 42, 43].

The article "Pakistan CO2 Emission Modelling and Forecasting: A Linear and Nonlinear Time Series Approach" was published in 2023. Journal: J Environ Public Health.

The simplest form of ETS [37, 42, 43] is given by

(8) $$\begin{array}{c} {\hat{x}}_{t+1\left|t\right.}=\beta x_{t}+\beta \left(1-\beta \right)x_{t-1}+\beta {\left(1-\beta \right)}^{2}x_{t-2}+\ldots , \end{array}$$

where *β*, 0 ≤ *β* ≤ 1, is the parameter for smoothing and *t* + 1 is the time for one-step-forward average forecast for the series *x*_1_,…, *x*_*t*_. *β* controls the rate of decrease in weights.

For ETS (A, N, and N), the additive model [37, 42, 43] is represented mathematically by

(9) $$\begin{array}{c} {\hat{x}}_{t}=F_{t-1}+\varepsilon_{t}, \end{array}$$

(10) $$\begin{array}{c} F_{t}=F_{t-1}+\beta \varepsilon_{t}, \end{array}$$

where (9) is the equation for the data and (10) is for the transition.

The ETS (A, N, and N) multiplicative model [37, 42, 43] is of the form

(11) $$\begin{array}{c} {\hat{x}}_{t}=F_{t-1}\left(1+\varepsilon_{t}\right),\\ F_{t}=F_{t-1}\left(1+\beta \varepsilon_{t}\right), \end{array}$$

where *ℱ*_*t*_ is the new level and *ℱ*_*t*−1_ is the previews level. *ε*_*t*_ is white noise with mean 0 and variance, *σ*^2^.

We, therefore, present the nonlinear machine learning time series model after thoroughly discussing linear time series models.

#### 2.2.2. Nonlinear Machine Learning Time Series Models

Here, we briefly discuss neural network autoregressive and multilayer perceptron nonlinear machine learning time series models.

*(1) Neural network autoregressive (NNAR) modelling approach*. A neural network autoregressive (NNAR) model is obtained when the lagged values of the time series are input to a neural network. NNAR (*p*, *r*) denotes *p* delayed inputs and *r* nodes. NNAR (*p*, 0) equals ARIMA (*p*, 0,0) without stationarity parameterization. The mathematical expression for NNAR (*p*, *r*) [36, 44–46] is of the form

(12) $$\begin{array}{c} h\left(y\right)=\beta_{0}+\overset{R}{\underset{r=1}{\sum }}\beta_{r}s\left(z_{k0}+\overset{p}{\underset{j=1}{\sum }}z_{rj}y_{j}\right), \end{array}$$

Model (12) can be constructed in two different stages, with the first being the activation *R*. Also, the hidden layer *B*(*r*) is computed as

(13) $$\begin{array}{c} B\left(r\right)=b\left(r\right)=s\left(z_{r0}+\overset{p}{\underset{j=1}{\sum }}z_{rj}y_{j}\right), \end{array}$$

where *r* = 1,…, *R* an d*y*_*j*_ = *y*_*t*−1,_ …, *y*_*t*−*p*_.*s* is a previously defined nonlinear activation function. Every *B*(*r*) acts as a unique transformation characteristic *b*_*r*_(*y*). Mathematically, the hidden layer,

(14) $$\begin{array}{c} h\left(y\right)=\beta_{0}+\overset{R}{\underset{r=1}{\sum }}\beta_{r}B\left(r\right), \end{array}$$

receives *R* instigations.

The article "Pakistan CO2 Emission Modelling and Forecasting: A Linear and Nonlinear Time Series Approach" was published in 2023. Journal: J Environ Public Health.

The NNAR model assumes a sigmoid function,

(15) $$\begin{array}{c} f\left(\omega \right)=\frac{1}{1+\exp\;\left(-\omega \right)}, \end{array}$$

used in the linear function translation of 0 probability to a probability of 1.

*(2) Multilayer Perceptron (MLP) Model*. The structure of the multilayer perceptron (MLP) model [47–50] is composed of the input layer, hidden layer, and output layer with limited nonlinear functions that are differentiable. In the MLP, information in the form of a nonlinear differentiable function is processed by artificial neurons from the input layer through the hidden layer to the output layer, yielding a response in the form of a disjointed feed-forward network algorithm. The mathematical expression of the MLP is given by

(16) $$\begin{array}{c} t\left(x\right)=k_{s}\left[\sum_{p=0}^{K}g_{1p}^{0}\left(k\sum_{n=0}^{N}g_{pn}^{i}c_{n}+d_{n}\right)\right], \end{array}$$

where *c*_*n*_, *d*_*n*_,*k*, *k*_*s*_, *t*(*x*), *g*_*pn*_^*i*^, and *g*_1*p*_^0^ are the network inputs, bias of the network, activation function of intermediate layers, output layer activation function, output signal, weights of the intermediate layer, and connections of output neurons, respectively.  Figure 3 shows the MLP model with a single hidden layer.

The RMSE and MAE will be used for all model comparisons.

R packages, forecastHybrid, forecast, Tplyr, caTools, T-series, nnet, TTR, and ForecastTB [51–57] were used for all modelling and forecasting.

## 3. Results and Discussion

From the time series plotted in Figure 3, the series is not stationary. We verified this by applying stationarity at the level (0) and found that the series is not stationary at the level (0). This means that the mean, variance, and covariance are not stationary over some time. This violation of nonstationarity was removed by taking the first difference of the series. We implemented the Dickey–Fuller (DF) test without drift, the Phillips–Perron (PP) test without drift, to verify whether our series is stationary or not, and the structural break (Chow test) [57] test to check whether there is a structural change in the series. The Chow test indicated that there is no structural change in the series as the *p* value is greater than 0.05. As a result, the series becomes stationary at the level (0). The output of these tests is given in Table 2 for the level (0).

The article "Pakistan CO2 Emission Modelling and Forecasting: A Linear and Nonlinear Time Series Approach" was published in 2023. Journal: J Environ Public Health.

From Table 2, the series is not stationary at the level (0), so we implemented a single differencing technique to make the series stationary. After making the series stationary, we searched for the best candidate model for the CO_2_ emission data by producing the correlogram of the differenced series. The visual autocorrelation (ACF) and partial autocorrelation (PACF) plots are presented in Figure 4.

In Figure 4, the ACF and PACF suggest that the estimated ARIMA model for modelling CO_2_ emissions includes two terms from the autoregressive (AR) part and one term from the moving average (MA) part. In the correlogram, the suitable ARIMA model for the series is ARIMA (4,1,7) since the lags of ACF and PACF are out of the boundaries on 5 and 7.

Using the complete dataset, we presented the visual single horizon forecast of the ARIMA, ETS, TBATS, naïve, NNAR, and MLP models in Figure 5, Figure 6, Figure 7, Figure 8, Figure 9, and Figure 10, respectively, to assess their visual performance. We traced the model performance visually to show the fitted versus the observed values. Figure 5, Figure 6, Figure 7, and Figure 8 show the visuals of linear time series modelling and forecasting, while Figure 9 and 10 show the visuals of the modelling and forecasting of nonlinear machine learning time series models.

We used the *nnfor* and *neuralnet* packages in *R* to perform the analyses for the nonlinear machine learning time series models. The packages adjust itself for the optimum number of parameters according to the behaviour of the series.

Although all models showed a similar trend as the original series (observed), the nonlinear machine learning time series models had a more closer trend compared to the linear time series models. This is an indication that the nonlinear machine learning models have superior forecasting qualities than the linear time series models.

The article "Pakistan CO2 Emission Modelling and Forecasting: A Linear and Nonlinear Time Series Approach" was published in 2023. Journal: J Environ Public Health.

Except for ETS and naïve models (Figures 6 and 8) which forecasted stable CO_2_ emissions in subsequent years, all other models forecasted increasing CO_2_ emissions in Pakistan in subsequent years. This trend is worrying and devastating and similar to that observed by Butt et al. [11].

We estimated the RMSE and MAE for both linear and nonlinear time series models to illustrate the numerical performance of our models.  Table 3 shows the RMSE and MAE estimates of all models using the complete dataset. From the table, we observe that RMSE values decrease in the order TBATS, naïve, ETS, ARIMA (4, 1, 7), MLP, and NNAR (1, 1), respectively, with the TBATS having the largest value and NNAR (1, 1) having the least value. For MAE values, the decreasing order is of the form TBATS, naïve, ETS, ARIMA (4, 1, 7), MLP, and NNAR (1, 1), respectively, with the TBATS having the largest value and NNAR (1, 1) having the least value. We noticed that both nonlinear machine learning time series models had smaller RSME and MAE values than all linear time series models, indicating their superiority to linear time series models. The NNAR (1, 1) model's least RSME and MAE values of 0.0007 and 0.0005, respectively, is a clear evidence that the machine learning nonlinear NNAR (1, 1) model possesses a superior forecasting quality and data assessment than the rest of the time series models. As a result, we utilized the NNAR (1, 1) model for forecasting CO_2_ emissions in Pakistan from 2019 to 2028. The forecast values as illustrated in Figure 9 show that CO_2_ emissions in Pakistan will be 1.048 metric tons per capita by 2028. This depicts a rapid increase in CO_2_ emissions from previous years. These results are in line with those of Aftab et al. [2] and Faruque et al. [3].

## 4. Conclusion

The present study related to forecasting and modelling CO_2_ emissions in Pakistan clearly warns that the current level of efforts made by the Government of Pakistan is not enough to capture the changes in climate change by reducing CO_2_ emissions. The increasing trend in emissions is a frightening and clear warning to policymakers. The increasing CO_2_ emissions is a serious threat to healthy living and fuels global warming vis-à-vis climate change. We call for pragmatic policy implementation by all stakeholders to bring finality to this alarming situation. To get a clearer picture of its increasing trend and to look for an accurate prediction of future CO_2_ emissions in Pakistan, this study employed a linear and nonlinear time series modelling approach to study CO_2_ emission data in Pakistan from 1960 to 2018, namely, ARIMA, naïve, TBATS, ETS, NNAR, and MLP. These linear and nonlinear time series models were used to forecast CO_2_ emissions for almost a decade. We utilized the complete data to present visual single horizon forecast for all models for easy visual comparison. Apart from the ETS and naïve models, which forecasted stable CO_2_ emissions in subsequent years, all other models forecasted increasing CO_2_ emissions in Pakistan in subsequent years. Our results reflected the findings of Ullah et al. [58]. Studies in China and India showed similar CO_2_ emission trends [15, 59, 60]. The RMSE and the MAE were used to check and assess the quality of the forecasting of models using the complete dataset. We observed that both nonlinear machine learning time series models had smaller RMSE and MAE values than all linear time series models, indicating their superiority to them. The NNAR (1, 1) model had the least RMSE and MAE values for the complete dataset. We, therefore, chose it as our best model for forecasting. Based on the forecasted value of the NNAR (1, 1) model, Pakistan's CO_2_ emissions will be 1.048 metric tons per capita by 2028. These results are in line with those of Aftab et al. [2] and Faruque et al. [3]. To achieve the targeted goal in the fight of reducing CO_2_ emissions, in order to accomplish the Paris Agreement of the UNFCCC, we propose that the Pakistan government should adapt the following:

- We should charge US$ 1000 per ton of CO_2_ emitted by companies and entities in every quarter of the year [61, 62]. This amount, which is set out by international authorities to curtail CO_2_ emissions, should be increased with time to discourage the use of high emitting fuels and encourage the use of low emitting ones. When this is initiated, it can reduce CO_2_ emissions by over fifty percent [61, 62].
- We should produce electricity from hydro, wind, and different sources with no emissions of CO_2_. This can reduce CO_2_ emissions in excess of seventy percent as well as make electricity cheaper [61].
- We should initiate rigorous planting of more trees, at least five million per year, in the populated areas of Pakistan as forest covers to absorb a greater chunk of emitted CO_2_ in the atmosphere. Studies reveal that five million trees in a particular area can absorb seventy percent of CO_2_ concentrates in the atmosphere in the area [61]. Therefore, this could reduce the concentration of CO_2_ in the atmosphere by over seventy percent of the recent value [61].
- We should provide, as a matter of urgency, incentives to companies, organisations, institutions, and households to come out with clean technologies or use technologies with no CO_2_ emissions or those with lower ones [61].
- We should fund more studies to develop clean and innovative technologies with less or no emissions [61]. This will go a long way to reduce emissions by over forty percent.

The article "Pakistan CO2 Emission Modelling and Forecasting: A Linear and Nonlinear Time Series Approach" was published in 2023. Journal: J Environ Public Health.

Our study can be used as a suggestion for forecasting CO_2_ emissions depending on different and dynamic settings. New policies for future purposes can be formulated and devised in light of this study. Our study can be extended to comparative analysis with other machine learning models using different activation functions.

## Figures and Tables

**Figure 1:** Time plot of CO_2_ in Pakistan from 1960 to 2018 (https://databank.worldbank.org/).

**Figure 2:** Steps involved in the Box–Jenkins methodology **(**source**:** Anvari et al. [37]).

**Figure 3:** Structure of multilayer perceptron (MLP) modelling with a single hidden layer.

**Figure 4:** Correlogram of the first difference of the series of CO_2_ emissions.

**Figure 5:** The ARIMA model for modelling and forecasting CO_2_ emissions.

**Figure 6:** The ETS model for modelling and forecasting CO2 emissions.

**Figure 7:** The TBATS model for modelling and forecasting CO_2_ emissions.

**Figure 8:** The naïve model for modelling and forecasting CO_2_ emissions.

**Figure 9:** The NNAR model for modelling and forecasting CO_2_ emissions.

**Figure 10:** The MLP model for modelling and forecasting CO_2_ emissions.

**Table 1:** Descriptive statistics of CO_2_ in Pakistan from 1960 to 2018.

Statistic	Estimate
Mean	0.572
Median	0.567
Maximum	0.982
Minimum	0.308
Standard deviation	0.191
First quartile	0.390
Third quartile	0.735
Skewness	0.259
Kurtosis	1.845

**Table 2:** The augmented Dickey–Fuller, Phillips–Perron, and structural break (Chow test) tests for CO_2_ emission data at the level (0).

Item	Estimate
Dickey–Fuller	−3.0238
Lag order	3
*p* value	0.161
Phillips–Perron unit root test	−9.6469
Lag order	3
*p* value	0.5404
Structural break test	
(Chow test)	
*p* value	1.00

The Phillips–Perron unit root test: 9.6469.

**Table 3:** RMSE and MAE estimates for linear and nonlinear time series models for the complete data.

Candidate models	RMSE	MAE
Naïve	0.0304	0.0236
ETS	0.0302	0.0232
ARIMA (4, 1, 7)	0.0239	0.0189
TBATS	0.0308	0.0240
NNAR (1, 1)	0.0007	0.0005
MLP	0.0020	0.0017

## Data Availability

The data consist of CO_2_ emissions in Pakistan from 1960 to 2018, available at https://databank.worldbank.org/.

## References

[1] United Nations (2021). Climate actions notes. https://www.unep.org/explore-topics/climate-action/what-we-do/climate-action-note/state-of-climate.html?gclid=Cj0KCQjwyt-ZBhCNARIsAKH1177SvL-qGAEaJyJtSDcYVKRAaMUh46G9VnwAloRnSPA8Wz5_aVTCKcEaAsoeEALw_wcB.

[2] Aftab S., Ahmed A., Chandio A. A., Korankye B. A., Ali A., Fang W. (2021). Modeling the nexus between carbon emissions, energy consumption, and economic progress in Pakistan: evidence from cointegration and causality analysis. *Energy Reports*.

The article "Pakistan CO2 Emission Modelling and Forecasting: A Linear and Nonlinear Time Series Approach" was published in 2023. Journal: J Environ Public Health.

[3] Faruque M. O., Rabby M. A. J., Hossain M. A., Islam M. R., Rashid M. M. U., Muyeen S. M. (2022). A comparative analysis to forecast carbon dioxide emissions. *Energy Reports*.

[4] Government of Pakistan (2021). Updated national determined contributions.

[5] Bokde N. D., Tranberg B., Andresen G. B. (2021). Short-term CO2 emissions forecasting based on decomposition approaches and its impact on electricity market scheduling. *Applied Energy*.

[6] Sun W., Li Z. (2020). An ensemble-driven long short-term memory model based on mode decomposition for carbon price forecasting of all eight carbon trading pilots in China. *Energy Science & Engineering*.

[7] Wu Q., Liu Z. (2020). Forecasting the carbon price sequence in the Hubei emissions exchange using a hybrid model based on ensemble empirical mode decomposition. *Energy Science & Engineering*.

[8] Yun P., Huang X., Wu Y., Yang X. (2022). Forecasting carbon dioxide emission price using a novel mode decomposition machine learning hybrid model of CEEMDAN-LSTM. *Energy Science & Engineering*.

[9] Eckstein D., Künzel V., Laura Schäfer L., Winges M. (2020). Global climate risk index 2020: who suffers most from extreme weather events? Weather-Related Loss Events in 2018 and 1999 to 2018.

[10] Iqair (2021). World’s most polluted countries and regions (historical data from 2018 to 2021). https://www.iqair.com/world-most-polluted-countries.

[11] Butt D., Myllyvirta L., Dahiya S. (2021). CO2 Emissions from Pakistan’s Energy Sector. https://energyandcleanair.org/wp/wp-content/uploads/2021/07/CO2-Emissions-from-Pakistans-Energy-sector_30_07_2021.pdf.

[12] Wu L., Liu S., Liu D., Fang Z., Xu H. (2015). Modelling and forecasting CO2 emissions in the BRICS (Brazil, Russia, India, China, and South Africa) countries using a novel multi-variable grey model. *Energy*.

[13] Pao H. T., Tsai C. M. (2011). Modeling and forecasting the CO2 emissions, energy consumption, and economic growth in Brazil. *Energy*.

[14] Chang H., Sun W., Gu X. (2013). Forecasting energy CO2 emissions using a quantum harmony search algorithm-based DMSFE combination model. *Energies*.

[15] Auffhammer M., Carson R. T. (2008). Forecasting the path of China’s CO2 emissions using province-level information. *Journal of Environmental Economics and Management*.

[16] Meng M., Niu D. X., Shang W. (2014). A small-sample hybrid model for forecasting energy-related CO2 emissions. *Energy*.

[17] Lin C. S., Liou F. M., Huang C. P. (2011). Grey forecasting model for CO2 emissions: a Taiwan study. *Applied Energy*.

The article "Pakistan CO2 Emission Modelling and Forecasting: A Linear and Nonlinear Time Series Approach" was published in 2023. Journal: J Environ Public Health.

[18] Pao H. T., Fu H. C., Tseng C. L. (2012). Forecasting of CO2 emissions, energy consumption and economic growth in China using an improved grey model. *Energy*.

[19] Amarpuri L., Yadav N., Kumar G., Agrawal S. Prediction of CO 2 emissions using deep learning hybrid approach: a Case Study in Indian Context.

[20] Lu I. J., Lewis C., Lin S. J. (2009). The forecast of motor vehicle, energy demand and CO2 emission from Taiwan’s road transportation sector. *Energy Policy*.

[21] Paravantis J. A., Georgakellos D. A. (2007). Trends in energy consumption and carbon dioxide emissions of passenger cars and buses. *Technological Forecasting and Social Change*.

[22] Rentziou A., Gkritza K., Souleyrette R. R. (2012). VMT, energy consumption, and GHG emissions forecasting for passenger transportation. *Transportation Research Part A: Policy and Practice*.

[23] Al-mulali U., Normee Che Sab C. (2013). Energy consumption, pollution and economic development in 16 emerging countries. *Journal of Economics Studies*.

[24] Wang T., Li H., Zhang J., Lu Y. (2012). Influencing factors of carbon emission in China’s road freight transport. *Procedia-Social and Behavioral Sciences*.

[25] Zhang C., Nian J. (2013). Panel estimation for transport sector CO2 emissions and its affecting factors: a regional analysis in China. *Energy Policy*.

[26] Lin F.-L., Inglesi-Lotz R., Chang T. (2018). Revisit coal consumption, CO2 emissions and economic growth nexus in China and India using a newly developed bootstrap ARDL bound test. *Energy Exploration & Exploitation*.

[27] Pao H. T., Tsai C. M. (2010). CO2 emissions, energy consumption and economic growth in BRIC countries. *Energy Policy*.

[28] Alam M. J., Begum I. A., Buysse J., Rahman S., Van Huylenbroeck G. (2011). Dynamic modeling of causal relationship between energy consumption, CO2 emissions and economic growth in India. *Renewable and Sustainable Energy Reviews*.

[29] Pao H.-T., Yu H. C., Yang Y. H. (2011). Modeling the CO2 emissions, energy use, and economic growth in Russia. *Energy*.

[30] Pao H.-T., Tsai C. M., Yang Y.-H. (2011). Multivariate Granger causality between CO2 emissions, energy consumption, FDI (foreign direct investment) and GDP (gross domestic product): evidence from a panel of BRIC (Brazil, Russian Federation, India, and China) countries. *Energy*.

[31] Ozcan B. (2013). The nexus between carbon emissions, energy consumption and economic growth in Middle East countries: a panel data analysis. *Energy Policy*.

[32] Zhang X. P., Cheng X. M. (2009). Energy consumption, carbon emissions, and economic growth in China. *Ecological Economics*.

[33] Cowan W. N., Chang T. Y., Inglesi-Lotz R., Gupta R. (2014). The nexus of electricity consumption, economic growth and CO2 emissions in the BRICS countries. *Energy Policy*.

The article "Pakistan CO2 Emission Modelling and Forecasting: A Linear and Nonlinear Time Series Approach" was published in 2023. Journal: J Environ Public Health.

[34] Bashir M. F., Ma B., Shahbaz M., Jiao Z. (2020). The nexus between environmental tax and carbon emissions with the roles of environmental technology and financial development. *PLoS One*.

[35] Box G., Jenkins G., Reinsel G., 4 (2008). *Time Series Analysis*.

[36] Daniyal M., Tawiah K., Muhammadullah S., Opoku-Ameyaw K. (2022). Comparison of conventional modeling techniques with the neural network autoregressive model (NNAR): application to COVID-19 data. *Journal of Healthcare Engineering*.

[37] Anvari S., Tuna S., Canci M., Turkay M. (2016). Automated Box–Jenkins forecasting tool with an application for passenger demand in urban rail systems. *Journal of Advanced Transportation*.

[38] Hyndman R. J., Anthanapoulous G., 2 (2018). *Forecasting: Principles and Practice*.

[39] RPubs by RStudio (2022). Why TBATS?. https://rpubs.com/chenx/tbats_notes.

[40] Basri K I., Sumitra I. D. (2019). Comparison of forecasting the number of outpatients visitors based on naïve method and exponential smoothing. *IOP Conference Series: Materials Science and Engineering*.

[41] Ahuja S., Kumar A. (2022). Expectation-based probabilistic naive approach for forecasting involving optimized parameter estimation. *Arabian Journal for Science and Engineering*.

[42] Arumugam R., Raji R. (2020). A Markov Model for Prediction of Corona Virus COVID-19 in India-A Statistical Study. *Xi’an Dianzi Keji Daxue Xuebao/Journal of Xidian University*.

[43] Jain G., Mallick B. (2017). *A Study of Time Series Models ARIMA and ETS*.

[44] Tealab A., Hefny H., Badr A. (2017). Forecasting of nonlinear time series using ANN. *Future Computing and Informatics Journal*.

[45] Benrhmach G., Namir K., Namir A., Bouyaghroumni J. (2020). Nonlinear autoregressive neural network and extended kalman filters for prediction of financial time series. *Journal of Applied Mathematics*.

[46] Hopfield J. J. (1988). Artificial neural networks. *IEEE Circuits and Devices Magazine*.

[47] Srinivasa K., Thilagam P. S. (2022). Multi-layer perceptron based fake news classification using knowledge base triples. *Applied Intelligence*.

[48] Deyasi A., Bhattacharjee A. K., Mukherjee S., Sarkar A. (2021). Multi-layer perceptron based comparative analysis between CNTFET and quantum wire FET for optimum design performance. *Solid State Electronics Letters*.

[49] Chai S. S., Cheah W. L., Goh K. L., Chang Y. H. R., Sim K. Y., Chin K. O. (2021). A multilayer perceptron neural network model to classify hypertension in adolescents using anthropometric measurements: a cross-sectional study in sarawak, Malaysia. *Computational and Mathematical Methods in Medicine*.

The article "Pakistan CO2 Emission Modelling and Forecasting: A Linear and Nonlinear Time Series Approach" was published in 2023. Journal: J Environ Public Health.

[50] Qureshi M., Daniyal M., Tawiah K. (2022). Comparative evaluation of multi-layer perceptron approach with conventional ARIMA in modeling and prediction of COVID-19 daily death cases. *Journal of Healthcare Engineering*.

[51] forecastHybrid (2020). Convenient Functions for Ensemble Time Series Forecasts. https://cran.r-project.org/web/packages/forecastHybrid/forecastHybrid.pdf.

[52] Bokde N. D., Yaseen Z. M., Andersen G. B. (2020). ForecastTB—an R package as a test-bench for time series forecasting—application of wind speed and solar radiation modeling. *Energies*.

[53] Tuszynski J., Dietze M. (2021). caTools: moving window statistics, GIF, Base64, ROC AUC, etc. https://search.r-project.org/CRAN/refmans/caTools/html/00Index.html.

[54] Trapletti A., Hornik K. (2022). Tseries: time series analysis and computational finance. https://cran.r-project.org/web/packages/tseries/tseries.pdf.

[55] Ripley B., Venables W. (2022). Feed-forward neural network and multinomial log-linear models. https://cran.r-project.org/web/packages/nnet/nnet.pdf.

[56] Ulrich J. (2021). TTR: Technical Trading Rules. https://cran.r-project.org/web/packages/TTR/TTR.pdf.

[57] Zeileis A., Leisch F., Hornik K., Kleiber C. (2002). Strucchange: an R package for testing for structural change in linear regression models. *Journal of Statistical Software*.

[58] Ullah S., Ozturk I., Usman A., Majeed M. T., Akhtar P. (2020). On the asymmetric effects of premature deindustrialization on CO2 emissions: evidence from Pakistan. *Environmental Science and Pollution Research*.

[59] Kirikkaleli D., Adebayo T. S. (2021). Do public-private partnerships in energy and renewable energy consumption matter for consumption-based carbon dioxide emissions in India?. *Environmental Science and Pollution Research*.

[60] Köne A. Ç., Büke T. (2010). Forecasting of CO2 emissions from fuel combustion using trend analysis. *Renewable and Sustainable Energy Reviews*.

[61] Newell R. G. (2021). Federal Climate Policy 101: Reducing Emissions.

[62] I M F B (2022). More countries are pricing carbon, but emission are too cheap. https://www.imf.org/en/Blogs/Articles/2022/07/21/blog-more-countries-are-pricing-carbon-but-emissions-are-still-too-cheap.

